The article "ECM-Mimicking Hydrogels Loaded with Bone Mesenchymal Stem Cell-Derived Exosomes for the Treatment of Cartilage Defects" was retracted in 2023. Reasons: signs of a paper mill; suspected computer-generated content; unreliable results or conclusions; concerns about the data.

# ECM-Mimicking Hydrogels Loaded with Bone Mesenchymal Stem Cell-Derived Exosomes for the Treatment of Cartilage Defects

**DOI:** 10.1155/2022/3450672

**Published:** 2022-11-03

**Authors:** Jiyun Cheng, Genxiang Rong, Ziqi Wang, Shencai Liu, Qinfeng Yang, Weilu Liu, Dongkun Zhang, Jianwei Li

**Affiliations:** ^1^School of Basic Medicine and Public Health, Jinan University, Guangzhou, Guangdong Province 510632, China; ^2^Department of Orthopedics, The First Affiliated Hospital of Anhui Medical University, Hefei, Anhui Province 230022, China; ^3^Department of Orthopaedics, Nanfang Hospital, Southern Medical University, Guangzhou, Guangdong Province 510515, China; ^4^Department of Thoracic Surgery, Guangdong Provincial People's Hospital/Guangdong Academy of Medical Sciences, Guangzhou, Guangdong Province 510080, China; ^5^Division of Orthopaedics and Traumatology, Department of Orthopaedics, Nanfang Hospital, Southern Medical University, Guangzhou, Guangdong Province 510515, China

## Abstract

It is well-established that treating articular cartilage injuries is clinically challenging since they lack blood arteries, nerves, and lymphoid tissue. Recent studies have revealed that bone marrow stem cell-derived exosomes (BMSCs-Exos) exert significant chondroprotective effects through paracrine secretions, and hydrogel-based materials can synergize the exosomes through sustained release. Therefore, this research aims to synthesize an ECM (extracellular matrix)-mimicking gelatin methacryloyl (GelMA) hydrogel modified by gelatin combined with BMSCs-derived exosomes to repair cartilage damage. We first isolated and characterized exosomes from BMSCs supernatant and then loaded the exosomes into GelMA hydrogel to investigate cartilage repair effects in *in vitro* and *in vivo* experiments. The outcomes showed that the GelMA hydrogel has good biocompatibility with a 3D (three-dimensional) porous structure, exhibiting good carrier characteristics for exosomes. Furthermore, BMSCs-Exos had a significant effect on promoting chondrocyte ECM production and chondrocyte proliferation, and the GelMA hydrogel could enhance this effect through a sustained-release effect. Similarly, *in vivo* experiments showed that GelMA-Exos promoted cartilage regeneration in rat joint defects and the synthesis of related cartilage matrix proteins.

## 1. Introduction

Since articular cartilage is an avascular tissue with limited intrinsic repair capacity, treating cartilage defects caused by trauma or illness remains challenging during clinical practice [1, 2]. To date, various treatments, including microfractures and arthroplasty, have failed to fully regenerate hyaline cartilage and restore its original mechanical properties due to the failure to generate sufficient tissue to restore damaged cartilage [3]. Damage to the articular cartilage can induce joint swelling and discomfort and precipitate the course of osteoarthritis, eventually leading to permanent full-thickness cartilage degradation and limb movement restriction [4]. Accordingly, a safe and effective treatment strategy for cartilage defects is warranted.

The article "ECM-Mimicking Hydrogels Loaded with Bone Mesenchymal Stem Cell-Derived Exosomes for the Treatment of Cartilage Defects" was retracted in 2023. Reasons: signs of a paper mill; suspected computer-generated content; unreliable results or conclusions; concerns about the data.

Mesenchymal stem cells (MSCs) are well-recognized to possess powerful immunomodulatory effects and tissue repair capabilities and have been widely used in cartilage-related diseases [5–7]. Indeed, significant inroads have been made in recent years, with reports that MSC transplantation can effectively promote the repair of cartilage damage by regulating the differentiation of MSCs into chondrocytes [8]. However, the efficacy of MSCs is limited by their poor cell survival at the injury site, the possibility of immunological rejection, and the uncertainty of differentiation direction after transplantation [9]. Overwhelming evidence substantiates that the therapeutic benefits of MSCs can be attributed to their paracrine mechanism, mostly involving the secretion of exosomes (Exos). Exos are cell-secreted vesicles 30–200 nm in diameter with similar functions to parental mesenchymal stem cells [10]. In addition, exosomes are easier to store and transport than cells, avoiding many limitations associated with cell transplantation, such as immunogenicity and tumorigenicity [11]. It has been shown that exosomes contain all kinds of lipids, proteins, and various noncoding RNAs, particularly miRNAs, which exert a regulatory role similar to their source cells by mediating cell-to-cell communication [12]. An increasing body of evidence from recently published studies suggests that exosomes can promote osteoarthritis repair and relieve pain by promoting cartilage regeneration and reducing inflammation [13]. However, the therapeutic effect of pure exosome therapy *in vivo* is limited, mainly due to insufficient local concentration and transient release of exosomes, which cannot guarantee a sustained effect. In addition, the repair and regeneration of cartilage damage needs a long healing time. Therefore, it is urgent to develop a good carrier to satisfy the need for local exosome release to maintain the bioactivity of exosomes and accelerate the repair of cartilage damage.

The advent of tissue engineering offers a promising avenue to resolve these problems. Given their decent biocompatibility and ease of modification, hydrogels are believed to be an appropriate material for delivering various active factors in most tissue engineering materials [14]. Gelatin methacryloyl (GelMA) is synthesized from gelatin by modification and contains numerous RGD (arginine-glycine-aspartic acid) and MMP (matrix metalloproteinase) target sequences involved in cell adhesion and are appropriate for cell remodeling [15, 16]. Due to GelMA's similarity with the extracellular matrix in some aspects and its adjustable mechanical properties, GelMA-based hydrogels have become suitable carriers for exosomes by changing the duration of light exposure, a technique widely used in nerve and growth plate injuries in children [17, 18]. Moreover, the GelMA hydrogel is endowed with injectable and chondroprotective properties after light exposure. However, few reports have been reported on cartilage injuries. Consequently, ECM (extracellular matrix)-mimicking GelMA hydrogels have huge prospects for clinical application to deliver exosomes to boost the repair of cartilage defects.

The article "ECM-Mimicking Hydrogels Loaded with Bone Mesenchymal Stem Cell-Derived Exosomes for the Treatment of Cartilage Defects" was retracted in 2023. Reasons: signs of a paper mill; suspected computer-generated content; unreliable results or conclusions; concerns about the data.

In this study, we synthesized a 3D (three-dimensional) porous hydrogel mimicking the ECM for delivering exosomes. The 3D porous structure of GelMA hydrogel enabled the retention and sustained release of exosomes secreted by bone marrow mesenchymal stem cells (BMSCs). Herein, we report a 3D hydrogel with ECM-mimicking properties that can be used to deliver bioactive exosomes to promote cartilage damage repair. The effects of long-term released exosomes in GelMA hydrogels on chondrocyte regeneration and cartilage defect healing were investigated *in vitro* and *in vivo*.

## 2. Materials and Methods

### 2.1. Isolation, Identification, and Staining of Exosomes from BMSCs (BMSCs-Exos)

BMSCs were collected by flushing the bone marrow cavity of 2-week-old rats' tibia and femur, as previously described [19]. The isolated BMSCs were put in a low-glucose DMEM (Gibco) mixture containing 10% serum and cultured at 37°C with 5% CO_2_ in a cell culture incubator. Passage 3 to 5 BMSCs (P3–P5) were used for subsequent experiments.

Gibco's low-glucose DMEM complemented with 10% exosome-free serum was used to culture the BMSCs. The supernatant was collected once the cells reached 50–60% confluency for ultracentrifugation. To separate live/dead cells and cell detritus, the supernatant was centrifuged for 10 minutes at 300 g, 3000 g, and 10,000 g. The exosomes at the bottom of the centrifuge tube were then resuspended in phosphate-buffered saline (PBS) and kept at −80°C after centrifugation at 100,000 g for 90 minutes. All the centrifugation procedures above were performed at 4°C.

Surface-labeled antibodies, such as CD9 (ProteinTech) and TSG101 (Abcam), were used to identify the collected exosomes. Transmission electron microscopy (TEM) and nanoparticle tracking analysis (qNa006E ® system, Izon Science) were used to examine morphology and size separately. Exosomes were stained with the red fluorescent dye PKH26 (Sigma-Aldrich) according to the manufacturer's instructions.

The article "ECM-Mimicking Hydrogels Loaded with Bone Mesenchymal Stem Cell-Derived Exosomes for the Treatment of Cartilage Defects" was retracted in 2023. Reasons: signs of a paper mill; suspected computer-generated content; unreliable results or conclusions; concerns about the data.

### 2.2. Establishment of an Exosome-Hydrogel System (GelMA-Exos)

5 g of gelatin (Gel, Sigma-Aldrich) was added to 50 ml of PBS solution and swirled until thoroughly dissolved at 50°C. The gelatin solution was then progressively added to 4 ml of methacrylic anhydride (MA, Sigma-Aldrich) at 0.5 ml/min, and the reaction was stopped after 3 h of continuous magnetic stirring at the specified conditions. The solution was dialyzed against clean water at 50°C for 6 days in a dialysis bag (12–14 kDa). The dialyzed solution was centrifuged at 2000 rpm for 10 minutes, and the supernatant was collected and lyophilized for 6 days in a freeze dryer to create a foamy methacrylic acid-modified gelatin sample (GelMA). GelMA was dissolved in heavy water (D_2_O) at 50°C, and the H^1^ NMR spectrometer was used to verify whether the modification was successful. The lyophilized The GelMA was dissolved in a photoinitiator Irgacure 2959 (Sigma-Aldrich) solution with a concentration of 0.5 w/v % to synthesize a prepolymerization monomer solution with a concentration of 10 w/v %. 200 *μ*g of exosomes were mixed well with 60 *μ*l of hydrogel solution and polymerized under UV irradiation (6.9 mW/cm2, 360–480 nm) for 15 s to obtain an exosome-hydrogel system (GelMA-Exos).

### 2.3. Material Characterization

Field emission scanning electron microscopy (FE-SEM, ZEISS) was used to examine the hydrogel's interior shape and structure. Frequency sweep of the hydrogel at constant strain (5%) with an Anton-Paar MCR 301 rheometer from 0.1 to 10 Hz to detect the storage modulus (G′) and loss modulus of the hydrogel (G″).

### 2.4. *In vitro* Degradation Test

Enzymatic degradation media were used to study the *in vitro* degradation of hydrogels. After being dissolved in 6 mL of PBS with 30 g/mL of collagenase type II (Sigma-Aldrich), the hydrogels were left to sit for an hour at 37°C. The remaining hydrogel was rinsed with PBS and its wet weights were recorded at each interval. By dividing the weight of the remaining samples by the weight of the original hydrogels, the percent degradation was computed.

### 2.5. Exosome Release and Uptake

Based on previous studies, cumulative and daily releases were evaluated using the BCA kit (Beyotime). In brief, the GelMA-Exos (*n* = 3) prepared above were incubated in PBS solution at 37°C. Supernatants were harvested on days 1, 3, 7, and 14, and free exosomes were detected by the BCA method. The total amount of exosomes minus the number of free exosomes in the supernatant was equal to the total amount of hydrogel-loaded exosomes.

The article "ECM-Mimicking Hydrogels Loaded with Bone Mesenchymal Stem Cell-Derived Exosomes for the Treatment of Cartilage Defects" was retracted in 2023. Reasons: signs of a paper mill; suspected computer-generated content; unreliable results or conclusions; concerns about the data.

To assess if the exosomes in the hydrogel exhibited phagocytic activity, chondrocytes were cocultured with GelMA-Exos for 1 d. Then the medium was removed, washed with PBS 3 times, and fixed for 20 min with 4% paraformaldehyde. The phagocytosis of exosomes was detected by laser confocal microscopy (Leica) (actin-Tracker Green (Beyotime) for the cytoskeleton and Hoechst 33342 (Beyotime) for the nucleus).

### 2.6. Biocompatibility Assessment

Chondrocytes were harvested from knee articular cartilage tissue of 2-week-old SD (Sprague–Dawley) rats as previously described [20]. The biocompatibility of the materials was assessed using live/dead staining, cell viability, and cell adhesion assays, respectively. First, 1 × 10^6^ chondrocytes were seeded on a 12-well culture plate and cocultured for 24 h with the samples of each group. The staining solution of PBS : Calcein-AM (Invitrogen): PI (Invitrogen) was supplemented to each group of samples in the ratio of 1 ml: 3 *μ*L: 5 *μ*L and incubated at 37°C for 20 min for laser confocal microscopy (Leica) observation. In addition, after coculturing the above chondrocytes with the samples of each group for 1, 3, and 7 days, the cell activity of each group was evaluated by measuring the absorbance at 450 nm with an enzyme-labeling instrument (BioTech) using CCK-8 reagent (Beyotime). Finally, chondrocytes at a density of 1 × 10^5^ were cocultured with the samples of each group for three days, then stained with Actin-Tracker Green (Beyotime) to evaluate cell adhesion in each group by a confocal microscope (Leica).

### 2.7. qRT-PCR Analysis

An RNA extraction kit (Omega) was used to extract total RNA, which was subsequently reverse transcribed into cDNA using the EVO-MLV RT kit (Accurate Biotechnology). LightCycler 480 SYBR Green Master Mix (TaKaRa) was used for the qRT-PCR analysis. The relative standard curve method (2-△△CT) was used to determine mRNA expression.  Table 1 shows the primer sequences.

### 2.8. Western Blotting

The samples were homogenized in RIPA lysis (CWBIO), including protease and phosphatase inhibitors (Thermo Fisher). After lysing on ice for half an hour, the supernatants were collected after centrifuging at 12,000 rpm for 30 minutes at 4°C. Then the BCA kit (Beyotime) was used to measure the total protein concentration. Equal amounts of protein were loaded on sodium dodecyl sulfate-polyacrylamide gel electrophoresis (SDS-PAGE) after loading buffer (Beyotime) was added to the supernatants. After the protein samples were deposited on the PVDF membrane (Thermo Fisher), they were blocked with 5% skimmed milk for an hour. The membranes were then treated overnight at 4°C with the primary antibodies specified in Table 2. The membranes were treated with secondary antibodies for one hour on the next day. Finally, immunoblots were examined using Thermo Fisher's enhanced chemiluminescence (ECL) kit. We cleaned the membranes three times in Tris Buffered Saline with Tween 20 (TBST) before each step. The quantitative analysis of proteins was analyzed using Image *J* software.

The article "ECM-Mimicking Hydrogels Loaded with Bone Mesenchymal Stem Cell-Derived Exosomes for the Treatment of Cartilage Defects" was retracted in 2023. Reasons: signs of a paper mill; suspected computer-generated content; unreliable results or conclusions; concerns about the data.

### 2.9. Immunofluorescence

After 30 minutes of fixation in PBS with 4% paraformaldehyde, the samples were treated for 10 minutes with 0.2% Triton X-100 (BioFroxx). Subsequently, a 3% bovine serum album (BSA, BioFroxx) was used to block these samples at room temperature for one hour. The primary antibodies were incubated at 4°C overnight; then, the secondary antibodies were employed for Hoechst (Beyotime) staining for 2 hours at room temperature. Before each step, we washed the samples three times with PBS. Finally, we observe the staining results under a confocal microscope (Leica). The antibodies are listed in Table 2.

### 2.10. Cartilage Defect Models

To study the effect of GelMA-Exos on cartilage repair, twelve eight-week-old SD female rats were randomly allocated into three groups: a simple injury group (Control), an Exos group, and a GelMA-Exos group. A mixture of 6 mg/kg pyrazine and 70 mg/kg ketamine were intraperitoneally injected to anesthetize these rats. Subsequently, the hairs on the left legs were shaved, and the skin was thoroughly disinfected with iodophor. The medial patella skin and muscle were cut under sterile conditions to expose the femoral condyle. Then a 15 G needle was used to create a central defect with a diameter of about 2 mm by drilling the articular cartilage. After treatment, the incision was sutured and disinfected again. Finally, they were kept in separate cages and given food and water freely.

### 2.11. *In vivo* Imaging, Histological Analysis, and Immunohistochemical Staining

In order to verify that GelMA-Exos can release exosomes *in vivo* for a long time, we detected the fluorescence signal intensity of exosomes by an animal *in vivo* imager 7 days after exosome implantation. Exosomes were stained with the red fluorescent dye PKH26 (Sigma-Aldrich) according to the manufacturer's instructions. The rats were slaughtered, and articular cartilage samples were taken after four weeks of treatment. The tissues were fixed in paraformaldehyde for 24 hours, then decalcified in 10% EDTA (pH 7.4) for 21 days before paraffin embedding and sectioning. The cartilage healing was examined using hematoxylin and eosin (H&E) and Masson staining after the sections were dewaxed in xylene, washed, and rehydrated with a series of graded ethanol. In addition, immunohistochemical staining was accomplished according to the standard protocols previously described. Information on the antibodies used is listed in Table 2.

The article "ECM-Mimicking Hydrogels Loaded with Bone Mesenchymal Stem Cell-Derived Exosomes for the Treatment of Cartilage Defects" was retracted in 2023. Reasons: signs of a paper mill; suspected computer-generated content; unreliable results or conclusions; concerns about the data.

### 2.12. Statistical Analysis

One-way analysis of variance (ANOVA) with Tukey's test was performed using GraphPad Prism 5 and SPSS 19.0. Experimental data were expressed as the mean ± standard deviation (SD). All experiments were repeated three times, and a *P*value <0.05 was statistically significant.

## 3. Results and Discussion

### 3.1. Characterization of BMSCs-Exos

The centrifuged exosomes were identified by particle size analysis, TEM, and Western blotting (Figure 1(a)). TEM showed that BMSCs-derived exosomes were round or oval and had a complete membrane structure with a size of about 100 nm (Figure 1(b)). Particle size analysis indicated that the diameters of BMSCs-derived exosomes ranged from 112 to 159 nm (Figure 1(c)), consistent with the literature [21]. A Western blot showed that these nanoparticles also expressed exosome surface-specific proteins CD9 and TSG101 (Figure 1(c)). These findings validated that exosomes produced from BMSCs were successfully obtained.

### 3.2. Synthesis and Characterization of GelMA-Exos

Two additional proton peaks belonging to methacrylamide (MA) groups in GelMA at 5.3 ppm and 5.5 ppm in the H^1^ NMR spectra of gelatin after methacrylic acid modification indicated that MA was successfully transferred to the gelatin molecule (Figure 2(b)) [22]. The storage modulus (G′) of GelMA-Exos was substantially larger than the loss modulus (G′) in the rheological property test, indicating that the synthesized hydrogel is a stable viscous solid (Figure 2(c)) [23]. Moreover, the storage modulus of GelMA-Exos was 968 ± 50 Pa, which meets the conditions for *in vivo* application (Figure 2(d)). Exos were uniformly dispersed on the hydrogel skeleton in SEM photos, validating that Exos were loaded into the 3D GelMA hydrogel (Figure 2(e)). Most importantly, we discovered that exosome release lasted 14 days and that over 80% of the exosomes were released from the hydrogel, which ensured the continuous release and sustained biological effects of exosomes at the cartilage injury site (Figures 2(f)–2(g)). Exos labeled with PKH-26 were also found to be scattered around the nucleus of the chondrocytes in immunofluorescence images, suggesting that Exos released from the hydrogel could be phagocytized by chondrocytes (Figure 2(h)).

### 3.3. Biocompatibility Assessment of Each Group of Samples

A better understanding of the biocompatibility of GelMA-Exos hydrogel is essential for treating cartilage defects. The live/dead assay revealed a large number of live cells (green) and a moderate number of dead cells in each group (red) (Figures 3(a)–3(b)). The CCK-8 assay revealed that chondrocyte proliferation increased with time (Figure 3(c)). On days 3 and 7, the GelMA-Exos group and the Exos group had considerably higher chondrocyte activity than the control group, indicating that exosomes could promote the proliferation of chondrocytes. In addition, there was a difference between the GelMA-Exos and the Exos groups on day 7, with the GelMA-Exos group having a considerably higher OD value than the Exos group, which could be ascribed to the GelMA hydrogel's sustained release action [24, 25]. Current evidence suggests that exos from MSCs can promote cell proliferation and migration while inhibiting apoptosis via the AKT and ERK signaling pathways [25]. Cytoskeleton staining revealed no significant difference between each treatment group and the blank group, and a large spreading area was observed in all cases, which indicated that the GelMA hydrogel had satisfactory affinity for chondrocytes (Figures 3(d)–3(e)). Interestingly, the excellent cell adhesion properties of GelMA have been attributed to its RGD and MMP-degraded sequence [26].

The article "ECM-Mimicking Hydrogels Loaded with Bone Mesenchymal Stem Cell-Derived Exosomes for the Treatment of Cartilage Defects" was retracted in 2023. Reasons: signs of a paper mill; suspected computer-generated content; unreliable results or conclusions; concerns about the data.

### 3.4. GelMA-Exos Promotes Repair of IL-1*β*-Injured Chondrocytes

To establish a cartilage injury in an *in vitro* model, we added IL-1*β* (10 ng/ml) (PeproTech, USA) to the chondrocyte culture medium for 1 day. A sample/IL-1*β*-treated chondrocyte coculture system was established, and the repair of chondrocytes in each group was detected by immunofluorescence staining, qPCR experiments, and Western blotting. Briefly, chondrocytes treated with IL-1*β* at a density of 1 × 10^4^ were cocultured with samples for 7 days, and the chondrocytes were repaired by quantifying catabolic (MMP-13) and anabolic markers (SOX-9, COL-2) in chondrocyte degradation. The expression of chondrogenesis-related genes SOX-9 and COL-2 in the GelMA group was higher than in the control group, but the difference was not statistically significant, indicating that the GelMA hydrogel mimicking chondrocyte ECM has a definite cartilage repair effect (Figure 4(a)) [27]. The GelMA-Exos and Exos groups had significantly higher SOX-9 and COL-2 expressions than the control group, whereas MMP-13 expression was significantly lower, indicating that BMSCs-derived exosomes protected chondrocytes from IL-1*β*-treated chondrocyte injury with the ability to promote chondrocyte repair [6, 28]. Furthermore, qPCR results revealed that the repair capacity of GelMA-Exos was more significant than the Exos group, indicating that the GelMA hydrogel produced a more significant sustained-release effect than exosome therapy alone. SOX-9 is widely thought to be one of the most important transcription factors in promoting chondrogenesis, as it regulates the production of chondrogenesis-related markers (type II collagen) and the development of the GAG matrix [29, 30]. MCSs-Exos have been documented to increase chondrogenesis, chondrocyte proliferation, and matrix production, primarily via noncoding RNAs such as miR-23b and miR-92a via MAPK, AKT, and ERK pathways [31, 32]. Consistent with the qPCR results, immunofluorescence staining and Western Blot showed that the GelMA-Exos group had the highest COL-2 protein expression and the lowest MMP-13 protein expression (Figures 4(b)–4(c)). Taken together, our results suggest that BMSCs-derived exosomes possess direct chondrogenic properties, while GelMA hydrogel yields a sustained-release effect to synergize exosomes.

The article "ECM-Mimicking Hydrogels Loaded with Bone Mesenchymal Stem Cell-Derived Exosomes for the Treatment of Cartilage Defects" was retracted in 2023. Reasons: signs of a paper mill; suspected computer-generated content; unreliable results or conclusions; concerns about the data.

### 3.5. GelMA-Exos Promote the Healing of Cartilage Defects in Rats

The establishment of the rat cartilage defect model and the implantation process of GelMA-Exos hydrogel are presented in Figure 5(a). *In vitro* degradation testing showed that the degradation rate of GelMA hydrogel was slow in PBS containing collagenase, and the doping of Exos did not affect its degradation rate (Figure S1). *In vivo* imaging of GelMA-Exos, seven days after implantation, showed that exosome signals were still detectable at the injury site but not with topical exosome treatment alone, indicating that the hydrogel can retain exosomes and enable sustained release (Figure 5(b)). Four weeks after establishing the animal model, the rat knee cartilage samples were collected for H&E and Masson staining (Figure 5(c)). HE staining showed new cartilage formation at the defect site. Collagen deposition and maturation were observed with Masson's trichrome staining. The staining results showed that the articular cartilage in the undamaged area was transparent and the surface was smooth and complete. Large cartilage defects and fractures were observed in the articular cartilage injury area in the control group, with little regenerated cartilage. The Exos group yielded a better repair effect than the control group, indicating that the Exos exert a protective effect at the injury site and promote cartilage regeneration. MSCs-derived exosomes have demonstrated unique therapeutic advantages in cartilage-related diseases in recent years. Zhang et al. discovered that mesenchymal stem cell-derived exosomes mediate cartilage regeneration by boosting chondrocyte proliferation and decreasing apoptosis via AKT and ERK signaling pathways [33]. Additionally, Yubao Liu et al. found that MSC-exosomes could promote chondrocyte proliferation and suppress apoptosis via the lncRNA-KLF3-AS1/miR-206/git1 axis [34]. Moreover, we found that the GelMA-Exos group exhibited better repair efficacy than the Exos group, which may be mainly attributed to the slow-release effect of the hydrogel. On the other hand, an increasing body of evidence suggests that GelMA is a gelatin-based hydrogel that mimics the natural extracellular matrix with tunable biological, degradable, and mechanical properties. It is considered a promising biomaterial for tissue engineering and regenerative medicine and has been applied to tissue engineering of many tissues, including bone, cartilage, and skin [35–37]. In conclusion, the above results corroborate that BMSCs-derived exosomes-loaded GelMA hydrogel can promote cartilage regeneration.

The article "ECM-Mimicking Hydrogels Loaded with Bone Mesenchymal Stem Cell-Derived Exosomes for the Treatment of Cartilage Defects" was retracted in 2023. Reasons: signs of a paper mill; suspected computer-generated content; unreliable results or conclusions; concerns about the data.

### 3.6. GelMA-Exos Promotes Cartilage Matrix Formation at the Injury Site

IHC was used to assess the expression of cartilage ECM-associated proteins (COL-2, SOX-9) in knee cartilage to better understand the relationship between cartilage extracellular matrix (ECM) and cartilage restoration (Figures 6(a)-6(b)). The Exos group exhibited significantly enhanced expression of SOX-9 and COL-2 at the injury site compared to the Control group, suggesting that BMSC-derived Exos may yield a chondroprotective effect and promote the expression of chondrogenesis-related proteins. Furthermore, compared to the Exos group, GelMA-Exos boosted the expression of COL-2, demonstrating that GelMA hydrogel enhanced the therapeutic effect of exosomes by sustained release and was consistent with the above results. Moreover, the study also proves that GelMA hydrogel can promote chondrocyte anabolism by supplying ECM essential for cartilage regeneration [15]. An increasing body of evidence suggests that exosomes derived from MSCs exhibit positive effects in regenerative medicine applications due to their ability to deliver regeneration-related RNAs, lipids, and proteins into target cells. MSCs-derived exosomes can mediate critical signaling pathways related to wound healing, such as AKT, ERK, STAT3, and IGF-1, promoting tissue regeneration [38]. On the other hand, besides the unique tissue repair ability of MSCs-derived exosomes, their potent anti-inflammatory effects cannot be ignored [39]. M1 macrophages infiltrate the injury site and release many proinflammatory molecules (such as TNF-, IL-1, and others) following cartilage damage. These inflammatory factors can persist and accelerate cartilage matrix deterioration. In addition, mesenchymal stem cells undergo aberrant differentiation in the inflammatory microenvironment, and chondrocytes begin to convert or dedifferentiate into fibroblast-like cells, resulting in fibrocartilage with poor mechanical qualities [40]. M2 macrophages also called wound repair macrophages, release a variety of anti-inflammatory chemicals such as Arg-1, IL-10, and others, which assist chondrocyte repair by suppressing MMP-13 expression and facilitating the repair of damaged chondrocytes [41]. It is widely believed that promoting the transformation of M1 macrophages to M2 macrophages during the inflammatory stage can aid in cartilage repair [42, 43]. In previous studies, we found that BMSC-derived exosomes carry various immune-regulating miRNAs, especially miR-199a, which can promote the metabolic balance of cartilage by regulating immunity [18]. In conclusion, we found that the GelMA hydrogel-loaded BMSCs-derived exosomes could promote the production of cartilage ECM-related proteins.

The article "ECM-Mimicking Hydrogels Loaded with Bone Mesenchymal Stem Cell-Derived Exosomes for the Treatment of Cartilage Defects" was retracted in 2023. Reasons: signs of a paper mill; suspected computer-generated content; unreliable results or conclusions; concerns about the data.

## 4. Conclusion

In this study, exosomes generated from bone marrow stem cells were loaded onto GelMA hydrogel to repair cartilage damage. The hydrogel can provide a sustained release of exosomes and enhance efficacy. *In vitro* experiments showed that the hydrogel loaded with exosomes had good biocompatibility and promoted the proliferation of chondrocytes as well as the ability to promote the synthesis of cartilage ECM. In addition, *in vivo* experiments showed that GelMA loaded with exosomes was beneficial in repairing cartilage injury in rats. This research broadens the therapeutic landscape for patients with cartilage injury in the clinic.

## Figures and Tables

**Figure 1:** Identification of bone marrow stem cells and their exosomes. (a) Schematic diagram of the extraction process of BMSCs-derived exosomes; (b) Micrograph of obtained nanoparticles by TEM; (c) Particle size analysis of the nanoparticles by qNano ® system; (d) Exosomes markers of CD9 and TSG101 by Western blot.

**Figure 2:** Characteristics of GelMA hydrogel loaded with exosomes. (a) Schematic diagram of GelMA hydrogel-loaded exosome synthesis; (b) NMR characterization of methacrylated gelatin; (c) Rheological analysis of GelMA-Exos hydrogel; (d) quantitative analysis of hydrogel rheological testing; (e) SEM image of GelMA-Exos hydrogel; (f) the daily release curve of exosomes (*n* = 3); (g) the cumulative release profile of exosomes for 14 days (*n* = 3); (h) exosomes loaded in the hydrogel were phagocytosed by chondrocytes.

**Figure 3:** Biocompatibility evaluation of each group. (a) Live/Dead analysis for each group after 1 day of cell culture; (b) quantitative analysis of live/dead assay (*n* = 3); (c) CCK8 assay of chondrocytes in each group (*n* = 5); (d) the cytoskeleton images showed the adhesion of chondrocytes after 3 days of culture in each group; (e) quantitative analysis of cell spread area (*n* = 3). ANOVA followed by Tukey's test was used for statistical analysis (^*∗*^*P* < 0.05, ^*∗∗*^*P* < 0.01, and ^*∗∗∗*^*P* < 0.001).

The article "ECM-Mimicking Hydrogels Loaded with Bone Mesenchymal Stem Cell-Derived Exosomes for the Treatment of Cartilage Defects" was retracted in 2023. Reasons: signs of a paper mill; suspected computer-generated content; unreliable results or conclusions; concerns about the data.

**Figure 4:** GelMA-Exos significantly alleviates the damage in IL-1*β*-treated chondrocytes. (a) chondrocytes were detected by qPCR after 7 days of culture in each group (*n* = 3); (b) Immunofluorescence detection of chondrocytes after 7 days of culture in each group; (c) quantitative analysis of fluorescence intensity of COL-2 and MMP-13 (*n* = 3). (d) Chondrocytes were detected by western blot analysis after 7 days of culture in each group (*n* = 3); (e) quantitative analysis of Western blot (*n* = 3). ANOVA followed by Tukey's test was used for statistical analysis (^*∗*^*P* < 0.05, ^*∗∗*^*P* < 0.01, and ^*∗∗∗*^*P* < 0.001).

**Figure 5:** GelMA-Exos significantly promotes the repair of knee articular cartilage injury in rats. (a) Schematic diagram of cartilage defect surgery; (b) *in vivo* imaging of rats seven days after GelMA-Exos implantation with or without hydrogel (PKH26-labeled exosomes can be observed in red); (c) H&E and Masson staining images of the injury site.

**Figure 6:** GelMA-Exos promotes the expression of chondrogenesis-related proteins at the injury site. (a) IHC staining of rat injury site; (b) Quantitative Analysis of IHC Staining in rat injured site (*n* = 3). ANOVA followed by Tukey's test was used for statistical analysis (^*∗*^*P* < 0.05, ^*∗∗*^*P* < 0.01, and ^*∗∗∗*^*P* < 0.001).

**Table 1:** Primer sequences of each gene.

Target	Forward	Reverse
COL-2	AACCCAAAGGACCCAAATAC	CCGGACTGTGAGGTTAGGAT
SOX-9	CGTGGTGACAAGGGTGAGAC	TAGGTGATGTTCTGGGAGGC
MMP-13	AGGCCTTCAGAAAAGCCTTC	GAGCTGCTTGTCCAGGTTTC
GAPDH	AGCCCAGAACATCATCCCTG	CACCACCTTCTTGATGTCATC

**Table 2:** Related information about primary antibodies.

Product Name	Species Reactivity	Dilution (cell/tissue)	Molecular weight (kDa)	Source
COL-2	Rabbit	1 : 200	142	Abcam, England
SOX-9	Rabbit	1 : 200	56	Abcam, England
CD9	Rabbit	1 : 1000	25	Proteintech, America
MMP-13	Rabbit	1 : 200	54	Abcam, England
TSG101	Rabbit	1 : 1000	46	Abcam, England

## Data Availability

All data used to support the findings of this study are included in the article.

## Supplementary Materials

Supplementary Materials Figure S1. *In vitro* degradation of GelMA and GelMA-Exos and in PBS with collagenase at 37°C over time (*n* = 4).
